# Based on the Auxiliary Effect of X-Ray in the Treatment of Severe Pneumonia in Children with Arterial and Venous Blood Gas

**DOI:** 10.1155/2022/5786630

**Published:** 2022-03-30

**Authors:** Hui Guo, Hua Zhang, Fuping Li

**Affiliations:** ^1^Department of Pediatric, Ji'an Matemal and Child Health Hospital, Jian 343000, Jiangxi, China; ^2^Department of Radiology, Ji'an Matemal and Child Health Hospital, Jian 343000, Jiangxi, China

## Abstract

Pediatric severe pneumonia clinical is a conceptual term for the diagnosis and treatment of pediatric clinical diseases. At present, domestic and foreign standards for clinical diagnosis of severe pneumonia, which is a childhood disease, are still inconsistent. At present, the first book of the main pediatric medical textbook in the society interprets the clinical definition of severe pneumonia in children as follows: severe pneumonia refers to pulmonary function in heart failure or other comorbidities in other important organs except the lung. This article is based on X-ray medical film and television examinations, through the analysis of arterial and venous blood gas in children with severe pneumonia to play a certain role in adjuvant therapy for children with pneumonia. Prospective clinical studies have found significant changes in the function of auxiliary coagulation and blood fibrinolysis indicators in patients with severe pneumonia in late childhood. The obvious difference between the pretreatment and the late-stage treatment for 1 week and the direct influence on the blood gas quantitative analysis and liver function of advanced patients provide a scientific basis for the diagnosis of typical advanced childhood severe pneumonia patients with adjuvant anticoagulant therapy. The data analysis of the clinical laboratory found that the blood coagulation and fibrinolysis functions of the typical patients with severe pneumonia in the typical late stage of childhood were significantly activated, and the anticoagulant antibody substances were significantly reduced, fibrinolytic coagulation inhibitors and anticoagulants are significantly increased, fibrinolytic activators are significantly reduced, and the body is in a procoagulant state for a long time. Adjuvant anticoagulation therapy through quantitative analysis of blood gas in patients can not only effectively increase the success rate of early treatment of typical late-stage severe pneumonia in children by 64.28% but also significantly reduce the inflammatory coagulation indexes of patients with late-stage severe pneumonia in children. The functions of coagulation, anticoagulation, and coagulation fibrinolysis have been significantly restored. The advantages of X-ray-based adjuvant treatment of severe pneumonia in children with arteriovenous blood gas are good contrast, clear imaging, and clear development of fine lesions or thick parts, and objective records are kept for comparison during review and consultation and discussion. The disadvantage is that the operation is more complicated, and it is not convenient to observe the activity function of the organ.

## 1. Introduction

Pneumonia bacterial infection disease is one of the most common pulmonary respiratory and nervous system diseases infection classification diseases, and many kinds of disease classification and diagnostic criteria have been developed clinically. It can be classified according to the type of pneumonia infection of various pneumonia-infected pathogens and can be divided into chronic pneumonia infection with bacterial viral tuberculosis pneumonia, viral pneumonia with bacterial tuberculosis pneumonia, and mycoplasmal viral tuberculosis pneumonia. It can also be classified according to the ways in which various types of pneumonia bacterial infections can be transmitted and can be divided into three types, pneumonia infectious tuberculosis pneumonia (community-acquired pneumonia, CAP) is obtained through adult community treatment, the hospital uses the treatment method to obtain pneumonia infectious tuberculosis pneumonia (hospital-acquired pneumonia, hap), and according to the inherent correlation of the human lung respiratory system different types of acquired pneumonia (ventilator-associated pneumonia, VAP) and so on. Regardless of the clinical classification, the diagnosis of pneumonia mainly depends on medical history, clinical manifestations, and imaging examinations, especially imaging examinations, which can distinguish pneumonia from other acute respiratory inflammations with similar symptoms. At present, the first choice for the diagnosis of pneumonia is a chest X-ray (CXR). In larger hospitals, digital radiography (DR) with better image quality is generally used; in smaller hospitals, ordinary chest radiographs may still be used due to conditions.

The lungs are vital respiratory organs that continue to keep in touch with the external environment, always face the threat of various environmental pathogenic factors, and are plagued by infectious diseases such as pneumonia. As one of the most common respiratory diseases, pneumonia is a high incidence and common disease at all ages. Its pathogen can come from the external environment or from the upper respiratory tract, which is the passage between the lung and the external environment. At present, the clinical imaging method for diagnosing pneumonia is mainly radiography, in which chest X-ray is often used as the first choice, and chest CT is considered the gold standard. Therefore, this article is based on X-rays to diagnose severe pneumonia in children and study the effect of blood gas analysis on the adjuvant treatment of severe pneumonia in children.

In recent years, blood gas analysis and determination have been carried out on the treated infants with pneumonia in a timely manner, and its role in the treatment is now discussed. Judging whether it is complicated by respiratory failure, infants with pneumonia complicated by respiratory failure often have a poor prognosis, so early diagnosis and timely rescue should be made. Observation confirmed that the changes of blood gas in infants and young children with pneumonia were related to the size of the lesions, the presence or absence of mutations, and whether viral pneumonia was secondary to bacterial infection.

This is because the incidence of severe pneumonia in children has increased and the mortality rate is high. The use of X-rays to diagnose and analyze blood to treat pneumonia has become an important method. Wen-bo has proposed the diagnosis of microcomputed tomography (MCT). Computer tomography uses a microfocused X-ray tube and a cone X-ray beam, which can display sample images from more than 360 angles. The same image sample can directly obtain the real isotropic and similarity of the smaller volume three-dimensional image, improve the three-dimensional spatial image resolution, and reduce the comprehensive use of radiation, but the application field is limited [1]. Hsinlj found the symptoms of children diagnosed with severe pneumonia in the early stage; CT clinical symptoms and examination pathological signs and analysis summary of CT examination are important clinical diagnostic and imaging methods for diagnosing severe pneumonia in children. Its clinical features are mainly that the area of the small intestine is thicker and more uniform, and the intestinal wall is gradually calcified. And on this basis, its cells appear unevenly into the tube wall and then into the soft tissue to form a larger thickness or round shadow of the mass. But this test can only be used for patients with chronic irritable bowel syndrome [2]. The cut-off value in the Van D statistical model is obtained from the ROC chart and subjected to discriminant analysis. The diameter and CT changes of the entropy and uniformity values are evaluated by a stepwise selection method. The critical values of the parameters are determined and the statistical model of the sample to evaluate the efficiency is analyzed and used for RECIST verification and discriminant analysis to create the Kaplan–Meier survival curve, but the diagnostic method is more complicated and difficult to apply to the actual situation [3]. Fu W reported a dilated X-ray framing camera based on a gated microchannel plate (MCP) and time dilation technique. The camera expands the electronic signal with a pulsed photocathode (PC) for high temporal resolution. The temporal resolution of the camera is characterized by short X-ray pulses produced by a laser beam focused on a flat iron target. The fringe raw images are obtained, and the experimental results show that the temporal resolution of the camera is better than 10 ps [4]. The Rohr J dual-source scanner is interested in the pathological type and clinical distance of severe pneumonia in children. The quantitative parameters of dual-source CT can indirectly reflect the pathological type of pneumonia and play an important role in the diagnosis of pneumonia. However, due to its expensive assembly cost, it is difficult to spread and use in a large area [5]. Stasevych M uses the grid-shaped sacroiliac combined with a radiofrequency neuron (PSRN) recommended by the study to treat severe pneumonia in children. CT-guided PSRN is safer and more effective in reducing the overall pain intensity in the treatment of arthralgia and pelvic pain in AS patients. The principle of improving the physical function and movement of the spine has been replaced by today's advanced equipment [6]. Wolff K D explored the clinical importance of chest computed tomography (CT) in the surgical treatment of pneumonia, but the extent of treatment is still limited [7].

The clinical pathology research report divides the two groups of children with typical severe pneumonia and acute patients into two groups, the first group is severe pneumonia benign, and the second group is severe pneumonia malignant group. Collect the serum ultrasound images of the two groups, respectively, and then compare the image characteristics (including the size, boundary, morphology of the nodule, the level of the mucosal echo halo within the nodule, the peripheral echo halo, the vertical and horizontal contrast, the calcification of the mucosal inside the nodule, the density change of the vascular flow pattern, and the chest X-ray examination), and the average data of children's blood gas density analysis step by step. The analysis data obtained by the patient are gradually collected by downloading the ACCESS software program data; after that, the accuracy of the statistical analysis results is analyzed through the SPSS19.0 software program, and the analysis results obtained by the patients are analyzed and displayed in the form of calculation of the average value of accuracy and ±standard deviation, respectively. For children's serum TSH and the statistical values of the image characteristics of the serum ultrasound image examination group, the *χ*^2^ test was carried out to determine the difference between the two groups of data. And to analyze and compare the accuracy difference data between the two groups of data, establish the regression analysis model of the logistic group of the nonspecific condition group, and use the ultrasonic forward step-by-step tracking analysis method to analyze the regression model step by step. Main functions of the advanced arterial blood gas analysis training model: this model is composed of a simulated hand model and an electronic blood circulation device. It has real blood flow, can palpate the radial artery, and feels real. Pulse speed and strength can be adjusted.

## 2. Principle and Overview

### 2.1. Pathology of Pneumonia

According to the different causes of pneumonia, tracheal pneumonia caused by various biochemical factors is referred to as similar bacterial tracheal pneumonia, viral tracheal pneumonia, mycoplasma tracheal pneumonia, fungal tracheal pneumonia, and various types of parasitic tracheal pneumonia. The types of tracheal pneumonia caused by different physical and chemical environmental factors are referred to as radioactive tracheal pneumonia, oil-like tracheal pneumonia, inhalation tracheal pneumonia, or allergic tracheal pneumonia, respectively. According to the different regions and scopes of the inflammatory lesions of thoracic pneumonia that may be involved, it can be subdivided into large-scale pneumonia similar to lobular nonbronchitis, lobular nonbronchitis pneumonia, and various types of pneumonia similar to segmental nonbronchitis [8, 9]. According to the main source of infection and nature of its pneumonia lesions, it can generally be roughly divided into serous, fibrinous, purulent, hemorrhagic, caseous, and various types of punctate granulomatous and edematous tracheal pneumonia. In clinical disease, it usually refers to the selection of the latest clinical names of pneumonia diseases that can accurately reflect the early characteristics of acute tracheal pneumonia lesions and the nature of lung inflammation lesions and give them accurate names in the hospital. The most common clinical symptoms of acute tracheal pneumonia in the period of vigorous onset of juvenile pneumonia are acute pneumonia accompanied by chronic pneumonia with small bronchitis, which can also be called pneumonia similar to lobular nonbronchitis. It mainly includes general bronchial pneumonia and interstitial pneumonia, both of which are common and frequently occurring clinical diseases. Generally speaking, chronic bronchial pneumonia is mainly a kind of purulent airway inflammation with acute pneumonia and lobular pneumonia as the main pathological unit. It is mostly caused by certain pathogenic bacteria such as *Staphylococcus pneumoniae* and *Haemophilus influenzae* bacteria, which have relatively strong or weak pathogenic immunity, and they are more likely to occur in the lower lobe and dorsal side. Interstitial pneumonia is mostly exudative inflammation, which is often caused by infections such as viruses and mycoplasma [10, 11]. Lobular pneumonia not only occurs in children but also occurs in the elderly, chronic patients, and other people with weakened immunity. In addition to lobular mucosal pneumonia in young adults, large lobular mucosal pneumonia is also common, which is mostly caused by f 1, 3, 7, and 2 types of lobular pneumonia and streptococcal infections that are highly infectious. It is an acute alveolar intima and diffuse mucosal exudative interstitial inflammation involving all large lobes of the lung; Figure 1 shows the real pathological diagram of human body weight pneumonia:

It is generally believed that the diagnosis of pneumonia mainly relies on medical history and physical examination. In fact, imaging examinations are widely used. A common belief is that patients with suspected pneumonia should undergo chest X-ray examination once they are admitted to the hospital [12, 13]. Sometimes sputum microscopy and sputum culture are also performed to understand the types of pathogenic bacteria to assist in the diagnosis and treatment of some complex and refractory cases. Because the lung tissue with air is considered to be the blind spot of ultrasound imaging, the imaging diagnosis of lung diseases, including pneumonia, mostly relies on radiological examinations, mainly chest X-ray and CT. Ultrasound has never been used clinically as a routine imaging examination item for pneumonia, and this situation still persists in China. In recent years, some scholars have also carried out lung MR examinations. The specific pathological classification of pneumonia and common diagnosis methods are shown in Table 1.

It is generally believed that chest X-ray is the preferred imaging method for patients with pneumonia, and chest CT is the imaging standard for the diagnosis of pneumonia. It is clinically recognized that the diagnostic value of chest CT is better than X-ray, but the former cannot completely replace the latter [14, 15]. The vast majority of literature believes that the diagnostic accuracy of CT is significantly higher than that of chest X-ray, but CT has the disadvantages of expensive, relatively long examination time, and relatively large radiation dose. And critically ill patients who cannot be moved cannot receive CT examinations but can only receive bedside chest radiographs. The medical examination process for pneumonia is shown in Figure 2:

Chest X-ray and CT have been used to diagnose pneumonia for a long time and are very mature diagnostic methods. At present, the focus of these two radiological examinations is for radiologists to reduce radiation dose by improving scanning methods and scanning parameters and to strike a balance between radiation dose and image quality. For clinicians and patients, it is the ionization damage to human tissues and related protection issues, as well as the feasibility of other nonradioactive imaging for the diagnosis of pneumonia [16, 17].

### 2.2. X-Ray Imaging Principle and Data Acquisition

X-ray is a commonly used medical imaging method. The basic procedure of X-ray imaging is to irradiate the inspected area with X-rays, then collect the radiation passing through the inspected area, and analyze the collected radiation dose. The collected and observed air radiation and energy have a certain positive correlation with the air density coefficient of the entire room. Imagine that the two parts illuminated by the sun are composed of small circles or rectangles (small circles or voxels) of the same ball size. The basic radiation amount irradiated on each different voxel is generally the same, but the remaining basic radiation amount is different after each different voxel of different voxel density is irradiated. The basic radiation attenuation coefficient is generally calculated from the increased radiation dose of the exposure residual [18, 19]. According to the basic attenuation coefficient of each voxel, the radiation attenuation value greater than X can be calculated and obtained. The calculation formula is as follows:

(1) $$\begin{array}{c} \text{X}=1000*\frac{\left(\mu_{\text{m}}-\mu_{\text{w}}\right)}{\mu_{\text{w}}}. \end{array}$$

Among them, m is the attenuation coefficient of a certain voxel, w is the attenuation coefficient of water, and the unit of the X-ray value is Hounsfield Unit (HU).

The delay time is analyzed, which made the algorithm in X-ray easier, so set the waiting time as Tback and rewind upper limit as TmaxBack:

(2) $$\begin{array}{c} \text{C}<16. \end{array}$$

Maximum avoidance index:

(3) $$\begin{array}{c} \text{Max E}=10. \end{array}$$

Maximum number of conflicts:

(4) $$\begin{array}{c} \text{MC}=16. \end{array}$$

Time slot:

(5) $$\begin{array}{c} \text{Slot}=\text{TbackN.} \end{array}$$

N is a positive integer between 0 and the upper limit of backoff:

(6) $$\begin{array}{c} \text{TMaxBack}=2^{\text{i}}-1,\text{i}\in \left(10,16\right). \end{array}$$

Similarly, the probability P of all nodes is not transmitting a data frame, the probability P of a single node transmitting P, the probability P of multiple nodes transmitting, etc. For the waiting time for any conflict to reach the desired value EB(i), when the number of conflicts is greater than 10, the expected value remains EB(10) unchanged; otherwise, it is EB(i). The estimated delay time is as follows:

(7) $$\begin{array}{c} \text{E}\left[{\text{T}}_{\text{i}}\right]={\text{P}}_{m}^{\text{i}}*{\text{P}}_{\text{r}}{\text{W}}_{\text{i}-1}. \end{array}$$

W_i-1_ represents the number of data arrival times before the i-th collision, so the total contention period delay time expectation can be expressed as

(8) $$\begin{array}{c} \text{E}\left[{\text{T}}_{\text{i}}\right]=\overset{\text{MC}}{\underset{\text{i}=0}{\sum }}\text{E}\left[{\text{T}}_{\text{i}}\right]. \end{array}$$

And the selection of the value of *i* in the backoff function is modified, for example, by selecting

(9) $$\begin{array}{c} \text{i}=\text{max}\left\{1,\text{MaxE}-\text{kC}+1\right\}. \end{array}$$

Or the following is taken:

(10) $$\begin{array}{c} \text{i}=\text{min}\left\{\text{TMback},2*\text{K}\right\}. \end{array}$$

The self-designed dynamic logarithmic BEB algorithm is adopted, and the K value adopts the dynamic logarithmic numerical method. And there are specific improvements to larger avoidance clues, specific settings:

(11) $$\begin{array}{c} \text{MaxE}=\text{fix}\left({\text{log}}_{2}\left(\text{N}\right)\right)\text{K}=\text{fix}\left({\text{log}}_{2}\left(\frac{\text{N}}{2}\right)\right). \end{array}$$

The backoff ceiling index is taken as:

(12) $$\begin{array}{c} \text{b}=\text{max}\left(1,\text{fix}\left({\text{log}}_{2}\left(\text{N}\right)-\text{k}*\text{i}+1\right)\right). \end{array}$$

The minimum is 2 and the maximum is 10; backoff upper limit time is as follows:

(13) $$\begin{array}{c} \text{TMback}=\left({\text{log}}_{2}\left(\text{b}+1\right)-1\right)*\text{T}\pm \text{slot.} \end{array}$$

Time slot:

(14) $$\begin{array}{c} \text{T}\pm \text{slot}=51.2*10\wedge \left(-3\right). \end{array}$$

The expected value of backoff index, when less than or equal to 10, is as follows:

(15) $$\begin{array}{c} \text{EB}\left(\text{i}\right)=\text{fix}\left(\left({\text{log}}_{2}\left(\text{b}+1\right)-1\right)*\frac{\text{T}\pm \text{slot}}{{\text{log}}_{2}\left(\text{b}+1\right)}\right). \end{array}$$

Otherwise,

(16) $$\begin{array}{c} \text{EB}\left(\text{i}\right)=\text{fix}\left(\left({\text{log}}_{2}\left(10\right)-1\right)*\frac{\text{T}\pm \text{slot}}{{\text{log}}_{2}\left(10\right)}\right). \end{array}$$

When the Vikj function monotonously increases *w* = 0, it will be a parameter when the Vikj function monotonously decreases:

(17) $$\begin{array}{c} \text{w}=1,\text{F}\left(\text{F}\in \left[0,\;1\right]\;\right). \end{array}$$

The equation guarantees

(18) $$\begin{array}{c} \text{x}\left[\text{isikj}\right]\text{new }\geq \text{ RVikj.} \end{array}$$

(19) $$\begin{array}{c} \text{x}\left[\text{isikj}\right]\text{new }\leq \text{x}\left[\text{isikj}\right]\text{old.} \end{array}$$

While complex images have high entropy, entropy can be defined as follows:

(20) $$\begin{array}{c} \text{entropy}=-\overset{{\text{N}}_{\text{i}}}{\underset{\text{i}=1}{\sum }}\text{P}\left(\text{i}\right)\log_{2}\text{P}\left(\text{i}\right). \end{array}$$

The basic idea of edge detection is to detect the edge points in the image first and then connect the edge points into contours according to a certain strategy to form a segmentation area. Since the edge is the dividing line between the target and the background to be extracted, the target and the background can be distinguished only by extracting the edge, so edge detection is very important for digital image processing. X-ray values penetrating all voxels in the radiation section can generate an X-value matrix and then obtain an X-ray image. Chest computed tomography is a method of using X-ray computed tomography to examine the chest. The characteristics of the X-value matrix are shown in Figure 3:

The thickness of the scan is usually 1 to 10 mm. The breast usually contains soft tissues and other organs belonging to the human body, such as the gastrointestinal tract and soft tissues, bones, fat, and various other soft tissues. The width and position of the window must be set differently. Different lung display parts need to pay attention to the width of the window. The width of the door in the window position is 400–500 HU, and the height of the window is 0–50 HU. It is suitable for displaying breast augmentation display of breast soft tissues such as the vertical and horizontal muscular atrial septal muscles of the upper and lower chest and abdomen on both sides of the human body. The window width is 1000–2000HU, and the window height is 600–800HU, which is suitable for display and intestinal scanning. The enhanced application of computerized chest tomography and various high-resolution new types of computerized chest tomography is the common surgical methods for the chest using computerized tomography. Simple X-ray scanning is the most common scanning method and does not inject contrast agent into the blood vessel. An enhanced X-ray scan is an X-ray scan that uses a contrast agent. In blood vessels, X-ray resolution has very high spatial resolution and density resolution and can clearly show the detailed structure of the tissue. The comparison of X-ray spatial resolution and density resolution factor is shown in Figure 4:

### 2.3. Principles of Blood Gas

The measurement of arterial catheter blood gas-related indicators is one of the commonly used clinical vital signs management and monitoring technical indicators, which involves many types of monitoring items, among which the more typical cases are PaCO_2_ and pH. PaCO_2_ can directly reflect the effect of detecting the patient's alveolar blood ventilation, and it is one of the important monitoring indicators for the clinical judgment of the patient's respiratory blood pH imbalance. Through the numerical monitoring of this monitoring index, it can be directly found whether there may be residual imbalances of respiratory carbon dioxide retention in the body of patients with lung disease. In this article, combined with the numerical analysis and monitoring of PH, the measurement results can directly assess whether there may be an imbalance of respiratory pH in patients with lung disease. At the same time, the analysis and determination of arterial catheter blood gas-related indicators is also one of the two key factors that clinically guide the clinical treatment and diagnosis of lung disease patients to predict the prognosis of the disease. The accuracy of analysis and measurement results of related technical indicators of arterial catheter blood gas indicators will directly affect its clinical value in practical medical applications. By analyzing the prognostic factors of patients' arterial catheter blood gas-related indicators analysis and measurement results, it is convenient to better formulate measures to take medical care and health management measures. Furthermore, it will gradually improve its related analysis indexes of arterial duct blood gas and the accuracy of the measurement results and give full play to its actual clinical application value for the measurement and analysis of arterial duct blood gas-related indexes.

It is well known that the X-ray beam generated by the medical X-ray generator is a mixed wave (white radiation) with rich frequency components. During X-ray inspection, the low-frequency components (i.e., low-energy X-ray photons) in such mixed waves may be absorbed in the interaction with the human body after passing through the human body for a certain distance. The lower the energy, the more likely the absorption. Some soft rays are absorbed even on the surface of the human body. These low-energy rays do not contribute to the X-ray image and only damage the human body. The more soft ray components are contained in the X-ray photon beam, and the medium (high) frequency high voltage power supply improves the X-ray image quality.

Early severe pneumonia in infants and young children is mainly an inflammation directly caused by bacterial infection of the respiratory tract in children. The disease mainly has the main characteristics of rapid onset, severe disease, and high fatality rate in children. Its main clinical symptoms are fever and dyspnea. Traditional oxygen therapy is currently an effective method for clinical treatment of the disease, but it is very easy to cause complications such as nasal mucosal ulcer, lung injury, and nasal septum injury in children, which limits its clinical application. The use of effective oxygen therapy measures is the key to improving the ventilatory function and ventilation status of infants and young children and controlling the progress of the disease. Warming and humidifying high-flow nasal catheter ventilation is a new type of oxygen therapy model based on the improvement of traditional oxygen therapy, which can effectively improve the tolerance of infants and young children. It can also assist in improving lung function and significantly improve the ventilation status of infants with severe pneumonia. The mechanism and effect of blood gas analysis on the treatment of severe pneumonia in children are shown in Figure 5.

Arterial catheter blood gas blood analysis is an important clinical diagnostic method that can quickly and accurately reflect the internal and external environmental health of critically ill children. The test results also directly affect the treatment decisions of the children's clinical nursing doctors, especially for children with critical symptoms. I personally recommend that nurses choose to use professional arterial blood gas detection tools for children and have reached a consensus on improving the accuracy of clinical test results. Clinical nurses in the pediatric department of acute and critical illnesses are more recommended to choose or use various professional arterial blood gas collection devices (choose professional arterial blood gas blood collection devices or use professional arterial vaccinations or puncture-type special arterial blood gas blood collection devices); 490 clinical nurses chose to use ordinary disposable arterial injectors for arterial blood gas sampling, accounting for 32.3%. Ordinary liquid blood inflatable syringes usually use hard plastic liquid inflatable injection tubes. Diffusion analysis will directly affect the blood inert gas that has entered this blood inert gas index and various other external chemical substances, resulting in the blood inert gas index dispersion analysis index being inaccurate. The main reason is that it affects the results of pH, PO_2_, and PCO_2_ in this blood gas index dispersion analysis, the standard bicarbonate (SB), actual bicarbonate (AB), residual alkali (BE), and extracellular residual alkali (BEecf) related to PO_2_ and PCO_2_. Therefore, in order to effectively ensure the accuracy of the results of the blood gas analysis of the commonly used arterial catheters, various large-scale specialized medical institutions specifically stipulate that nurses should strictly follow the norms to use a new type of more professional and commonly used arterial stent catheter blood gas venous blood analysis and blood sampling device detection and identification device [20, 21].

In addition, when using a disposable blood metering syringe or a new type of arterial catheter blood gas blood sampling instrument that is commonly used as a common arterial small plate blood gas catheter blood quantitative analysis test result to identify specimens, one of the 60.5% of nurses would recommend the use of a freeze-dried saline solution containing calcium and heparin sodium for blood rinses. The experimental results show that the salt of heparin sodium has strong physical and chemical substance selectivity and chemisorption to the negative ion heparin calcium sodium of yang and yin. It will directly result in that other nurses exchange the commonly used anticoagulant with the sodium heparin calcium in the blood for ion exchange, affect the exchange of calcium and heparin sodium, magnesium, calcium, and heparin sodium magnesium, and use quantitative detectors and other methods to test the certainty and accuracy of the results. Therefore, a nurse is specifically recommended to use a lyophilized salt and a lyophilized salt-containing heparin sodium, or a self-filling, disposable type containing other commonly used anticoagulants, or nonuse of the new safety-type common arterial catheter blood gas blood sampling instrument testing equipment. The preset and nonused arterial catheter blood gas blood sampling devices are also authoritative international arterial blood sampling technical guides, specifically stipulating that the equipment is recommended for use by a nurse [22, 23].

## 3. Experiment and Design

### 3.1. Design of Experimental Control Group

Children with severe pneumonia present with obvious pathological changes such as pulmonary respiratory tract inflammation, sputum secretions, and high-concentration reactions in the respiratory airways. In addition, the children also have increased glucocorticoid-1 in plasma cells and decreased nitric oxide cell synthesis protein; platelets synthesize granule membrane protein-140; the platelet-activating factor is significantly increased; the ratio of thromboxane A2 to thromboprostaglandin 2 is imbalanced. These abnormalities may indicate that pneumonia is beneficial to the damage of the vascular mucosal endothelial layer and the exposure of thrombus collagen under the endothelium, which directly activates the platelets and prothrombin oxidase in the lungs of the children and leads to a hypercoagulable state. The results of clinical studies such as Lin Chunwang [24] showed that there is a hypercoagulable state in the lungs of children with severe pneumonia and causes the formation of acute microthrombosis in the lungs, D-deoxydimer (D-Dimor, dd) increased significantly, and the activity of AT-III decreased significantly. The activation time of thrombin kinase (TT) and the activation time of thrombin prokinase (APTT) in some children were significantly shorter than those in the normal infection control group, and the intra-arterial thrombin oxidase saturation (SaO_2_) was significantly reduced. The prothrombin activation time (PT), activation time (APTT), TT, and DD of some children with normal infection were significantly higher than those of the normal infection control group. Although it is in the normal infection range, it is lower than the normal infection control group. The large differences in the results of the two clinical studies may be closely related to the severity of the lung infections and the duration of the disease in the two study subjects [25].

Adrenal secretory function, side effects of c-cell metabolism, and venous blood protein were analyzed by antibodies and venous blood flow from the blood flow monitoring of the arteries in the peripheral ventricle. The two methods of testing one ELISA at a time were used to test one PAl-1 twice. Both the normal control group and the long-term control group were physical examiners from the physical examination group of the health clinic of our hospital in Beijing in 2015. He asked for a health examination of peripheral upper peritoneal venous blood after fasting at 6 : 30 in the morning [26]. This prospective clinical study has obtained changes in the concentration of liver coagulation and other fibrinolytic liver functions in patients treated with chronic pneumonia in this community. The difference between the concentration before treatment and the patient's 1 week after treatment has an important impact on the analysis of the liver function of the treated patient's liver blood gas map. Moreover, the treatment of patients who may have other severe liver damage and whether it may affect other coagulation and fibrillary functions provides a scientific basis for diagnosing early pneumonia diagnosis and whether it is suitable for the application of other conditions anticoagulant treatment methods.  Figure 6 shows the comparison of blood gas factor index data between children with severe pneumonia and the normal control group.

The research subject is a late-stage community resident who is hospitalized in the late-stage community and the patients with chronic pneumonia are the main investigation and research objects. The prospective big data analysis research is based on the analysis of the obvious damage to the overall liver function of the patient with chronic pneumonia obtained by a resident in the community at the time of the disease; the obvious difference between the prognosis before treatment and the late prognosis at 1 week of treatment, the objective analysis of the late systemic local blood gas structure of a severe late-type patient, and the direct damage to liver function; and whether a severely late-type patient undergoes significant changes in the degree of systemic liver function damage when receiving a viral infection in the late stage and whether it can directly affect the overall liver function of a severely late-stage patient, such as systemic local coagulation, anticoagulation, and local coagulation and fibrinolysis. A scientific basis is provided for whether the late treatment of severely ill late-type patients with chronic pneumonia in the advanced community who need long-term use of short-acting anticoagulants can become a direct treatment and diagnosis target so as to effectively help control or shorten the clinical recurrence period and course of severely ill advanced patients with chronic pneumonia in the advanced community, improve the prognosis, and reduce the late mortality of severely ill patients.

### 3.2. Experimental Equipment and Objects

#### 3.2.1. Research Object

A total of 252 cases of children with severe pneumonia in children and children in the outpatient of the department of vascular medicine of a children's hospital were counted at the same time. There were 152 cases from 36 months to 6 years old at the same time and 200 cases over 6 years old. The relationship between the number of patients with severe pneumonia and their age is shown in Figure 7:

The basic criteria for the clinical diagnosis of acute severe pneumonia in children, the full text refers to the diagnosis concept of severe pneumonia in children in the WHO Children's Acute Pneumonia Respiratory Bacterial Infection Prevention and Control Program, and the diagnostic criteria for other chronic diseases in children refer to the 7th edition of Zhufutang Pediatrics. Chemical clinical diagnosis of pathogenic bacteria in sputum culture: based on the clinical chemistry diagnosis method, the sputum of children who meet the chemical screening was separated twice to isolate the same other pathogenic bacteria. Specimen identification of pathogenic strains of typical mixed acute infection: during the same period, two consecutive samples were analyzed and detected to isolate other different pathogenic bacteria, and the child was determined to be a typical mixed acute infection pathogenic strain.

The experimental equipment is shown in Table 2:

Short analysis time: 17 critical parameter results are obtained in 35 seconds, and timely treatment plans are given to patients. Short cycle time: sample testing can be performed at any time, and the timeliness of sample testing will not be affected by maintenance. Automatic quality management (AQM) system monitors the entire inspection system and random errors in real time through calibration, quality control, and internal inspection of the system and corrects them in time.

### 3.3. Experimental Operation

The patient was admitted to the hospital for diagnosis, the chest patient was checked immediately after admission this week, and two X-ray lasers and radiographs were taken in the chest and abdomen to determine the location where the peripheral malignant lesion may occur and the extent of the lesion. Blood samples of sputum coagulative leukemia from peripheral lesions were collected and blood smears, blood analysis, and culture were performed. By combining the clinical symptoms of peripheral lesions and performing laboratory tests based on clinical examination signs, the peripheral lesions were diagnosed as children with severe pneumonia, and the main fluids were taken immediately for blood tests. After blood analysis and testing, the main blood tests for urine and liver routine, four items of coagulation, DD, AT-III, and four analyses of blood gas concentration were performed. The two main detection materials and ELISA methods were used to detect renal tubular coagulation function and CRP, respectively. The specific operation flow diagram for detecting the content of the above body characteristics is shown in Figure 8.

Taking the concentration of the standard substance as the abscissa, draw a standard curve on logarithmic graph paper, and find the corresponding concentration range on the standard curve. The specific operation steps for detecting t-PA in human blood and the comparison of inflammatory indexes between each group are shown in Table 3.

Using clinical retrospective medical history analysis method, the inspection indicators are as follows:

1. Examination of the occurrence of complications in children
2. Auxiliary medical examination of children, mainly including blood routine, blood meteorological analysis and blood electrolytes, blood coagulation and lung function at discharge, imaging, pathogen culture detection (mainly including searching for negative sputum cells, virus receptor antigens in the respiratory tract, blood and mycoplasma virus antibody culture tests, and negative sputum cell culture), and the results of drug susceptibility detection mainly used for pathogenic bacteria
3. Combination therapy, including antibacterial hormone drug combination therapy, hormone drug therapy, supportive drug therapy, and the use of medical mechanical ozone ventilators
4. The prognosis of cure, mainly including the prognosis of cure, improvement, giving up, and finally death

## 4. Experimental Data Processing and Results

### 4.1. Data Collection and Processing

SPSS 17.0 statistical data analysis application software was used for statistical data analysis of the importance of statistical data samples of independent measurement laboratories. Before conducting important statistics on the data samples of independent measurement experiments, it is first necessary to carry out a comparison test of normality and variance. Those conforming to the positive and the same negative count standard deviation distribution are represented by the function formula that the variances are all mean ± standard deviation (*x* ± *s*). The comparison of statistical means of variance between two groups generally mainly adopts the comparison test of variance *t* and negative *t* variance, and the comparison of statistical means of variance between multiple groups generally mainly adopts analysis of variance. Different from those who just fit the normal count standard deviation distribution, the variance is the median (including the three-quarter digits and the gap in the middle). The [m(Q)] function formula is an example to show that the statistical standard value positive rank and variance comparison test of two different independent statistical experimental data samples is performed. The standard value X2 test is generally used for the variance of the negative count measurement data. The high accuracy of *p* < 0.05 is an important statistical data analysis and practical significance. The detailed data are shown in Figure 9:

Severe pneumonia in children often occurs in heart and lung organs and local lung function and nervous system heart failure (multiple organ failure, MOF), and the early high incidence is common in June to December. Moderate viral A leukemia encephalopathy is more common in the early stage of the disease from 28 days to June. The comparison of coagulation and fibrinolysis indexes among patients is shown in Table 4.

## 5. Results

Of the 252 cases of acute high-risk severe pneumonia in all children, only (121/252) two cases have high-risk severe disease risk factors. These high-risk severe diseases have a total of 161 cases. Among them, acute pediatric cardiovascular and nervous system diseases, malnutrition, brain dysplasia (155/252) cases have high-risk clinical complications in the occurrence of the disease, and there are 231 cases of high-risk clinical complications of these diseases. Among them, acute pediatric respiratory failure and acute pediatric heart failure patients with severe diseases are the main clinical high-risk complications, accounting for 62.3% (144/231). The data of each part of the inspection method is shown in Figure 10.

Compared with the normal combined control group, patients with early symptoms of B pneumonia also reflect the abnormal blood index of the function of human blood clotting cells. The coagulation combined enzyme activation time (TT) has been shortened a lot (*p* < 0.02). The clinical symptoms of patients with type B pneumonia at the initial stage of blood coagulation treatment were that the partial pressure of oxygen (Pa0_2_) and the saturation of intra-arterial coagulation of oxygen (S02) were significantly lower than those of the normal combined control group (*p* < 0.02) and lactic acid (lac) was significantly increased (*p* < 0.02). Before the rehabilitation of patients with advanced pneumonia, the levels of blood pressure (PaCO_2_) and bicarbonate (HC0_3_-) were significantly different between the group using of carbon dioxide lysing enzyme to break down blood pressure (PaCO_2_); in the normal treatment control group, there was no significant statistical fact (*p* > 0.05). After rehabilitation treatment, both were significantly lower than those in the normal treatment control group (*p* > 0.05). However, after diagnosing pneumonia in children with severe pneumonia based on X-rays, the targeted arterial and venous blood gas analysis and treatment of the children have increased the treatment rate by 64.28%.

## 6. Conclusion

This article mainly adopts a prospective fasting controlled clinical study test method, examining the patients before and after fasting and the hospital health doctor group before and after comparison. In 252 children with severe pneumonia, based on chest X-ray radiation, the entire body of the patient was examined by optical video imaging of the chest and checked immediately afterward (groups *b* and c). And on the 7th day (group c) at 6 am in the morning, coagulation and urine routine test, four items of coagulation, and D-dimer were taken from the peripheral blood vessel and venous blood flow test piece on an empty stomach (antithrombin-Ill (AT-III), liver function, adrenal function, CRP, blood protein). Taking the peripheral arterial blood flow examination film and blood gas data analysis, compared with the normal oxygen inhalation control group, the main body kidney and liver functions of children with severe pneumonia and poor children have not suffered severe damage. It is not important to affect the hemostatic, anticoagulant, and inhibitory functions of coagulation protein fibrinolytic complex enzyme. One of the shortcomings of the current research of this research topic is that the duration of the research work of this topic is relatively short and the sample size is relatively small. In the future continuous research, the sample size in this study should be larger, and further study is warranted to understand the characteristics of clinical medical pathology, etiology, and drug resistance of children with acute severe pneumonia in the society. Moreover, in the future, its clinical medical background to analyze the factors that affect it and its pathological changes should be analyzed, the direct causal relationship between children with acute severe pneumonia and poor prognosis in children examined, high-risk factors identified, clinical evidence for the early diagnosis and prevention of severe pneumonia provided, and the rational clinical selection of antibiotics guided.

## Figures and Tables

**Figure 1:** Pathological diagram of severe pneumonia.

**Figure 2:** Medical examination process for pneumonia.

**Figure 3:** Schematic diagram of the characteristics of the X-value matrix.

**Figure 4:** Comparison of X-ray spatial resolution and density resolution factor.

**Figure 5:** The mechanism and effect of blood gas analysis in the treatment of severe pneumonia in children.

**Figure 6:** Blood gas factor index of children with severe pneumonia and normal control group.

**Figure 7:** The relationship between the number of severely ill children and their age.

**Figure 8:** Operation flowchart for detecting PAl-1 in human blood.

**Figure 9:** The data graph of the patient's and children's prevalence.

**Figure 10:** Examination method data for each part of the patient.

**Table 1:** Classification of pneumonia and common diagnostic methods.

Types of pneumonia	Diagnosis method
Mycoplasma pneumonia	X-ray
Chlamydia pneumonia	CT
*Staphylococcus aureus* pneumonia	MR
Adenovirus pneumonia	X-ray

**Table 2:** Details of the experimental equipment.

Equipment name	Model	Origin
Blood gas analyzer	Raydu ABL-520 blood gas analyzer	Denmark
Lactic acid determination	Raydu ABL-520 blood gas analyzer	Denmark
Blood routine	Sysmex SF-3000 automatic blood cell analyzer	America
Coagulation	Diagnostica Stago coagulation analyzer	America
Low-temperature centrifuge	Beckman Coulter	America

**Table 3:** Comparison of inflammatory indexes between groups.

Group	WBC	GR (%)	PLT	CRP (mg/L)
A	10.12 ± 6.25	65.26 ± 12.26	312.58 ± 128.69	110.25 ± 76.58
B	8.26 ± 2.51	62.52 ± 10.36	325.26 ± 118.25	9.25 ± 8.14

**Table 4:** Comparison of coagulation and fibrinolysis indexes between groups (*x* ± *s*).

Test items	Group A	Group B	Group C
PT (s)	13.52 ± 1.06	13.58 ± 0.58	14.58 ± 1.69
APTT (s)	35.29 ± 1.25	39.52 ± 6.54	35.66 ± 4.89
TT (s)	17.25 ± 1.82	15.78 ± 4.89	15.89 ± 2.58
FIB (g/L)	3.12 ± 0.48	6.41 ± 2.18	5.10 ± 1.57

## Data Availability

The data that support the findings of this study are available from the corresponding author upon reasonable request.
